This article has been retracted.

# Feasibility Analysis of 3D Printing-Assisted Pedicle Screw Correction Surgery for Degenerative Scoliosis

**DOI:** 10.1155/2022/4069778

**Published:** 2022-09-06

**Authors:** Xuanhuang Chen, Xiaoqiang Gao, Feng Zheng, Haibin Lin

**Affiliations:** Department of Orthopedics, The Affiliated Hospital of Putian University, Putian, Fujian 351100, China

## Abstract

**Objective:**

To explore the feasibility of 3D printing-assisted pedicle screw correction surgery for degenerative scoliosis.

**Methods:**

From January 1, 2015 to January 31, 2020, patients with degenerative scoliosis who received corrective surgery in our hospital were retrospectively analyzed. Patients were grouped based on the fixation methods. Patients in the control group received traditional pedicle screw internal fixation, while those in the study group received 3D printing-assisted pedicle screw fixation. The therapeutic effects were compared.

**Results:**

There were 78 cases in the control group and 82 cases in the study group. There were no significant differences in scoliotic Cobb's angle, pelvic incidence-lumbar lordosis (PI-LL), VAS score, JOA score, social function, physical function, role function, or cognitive function between the study group and the control group before the surgery, but there were differences in the above parameters between the two groups after surgery. The incidence of postoperative complications in the study group was also significantly lower in the study group.

**Conclusion:**

3D printing-assisted pedicle screw correction surgery provides a strong 3D correction force with reliable effect and fewer complications, and is a good treatment choice for degenerative scoliosis.

## 1. Introduction

In degenerative scoliosis, the deformity of the spine is three-dimensional (3D) and rotational due to the progression of the lesions in the vertebrates. The Cobb angle is characteristically over 10°. The lesions initiate as asymmetric degeneration in the disc and joints, producing asymmetric loading and subsequent deformity. The symptoms include pain with neurological deficits. Nonsurgical treatment includes medication and physical therapy. Alternatively, epidural injections for selective nerve root blockade may be used [1, 2]. In patients with uncontrollable pain or neurological deficits, the purpose of surgery is to decompress neurons by repairing, modifying 3D deformities, and stabilizing vertebrate balance. This study investigated the feasibility of 3D pedicle screw correction surgery for degenerative scoliosis.

## 2. Materials and Methods

This study included patients who received degenerative scoliosis and correction surgery at our hospital from January 1, 2015, to January 31, 2020. The ethics committee of our hospital approved this study. All included patients and their families were informed of the study and actively signed informed consent. The inclusion criteria were: (1) Clinically confirmed degenerative scoliosis; (2) corrective surgery required; and (3) normal cardiopulmonary function. The exclusion criteria were: malignant disease, mental illness, drug allergy, any previous treatment of degenerative scoliosis with surgeries or medications, chronic diseases that need long-term medication such as hypertension, diabetes, etc., or lost-to-follow-up.

### 2.1. Methods

All patients received frontal and lateral X-ray photography of the whole spine before surgery for determination of the patient's scoliosis and rotation; left and right refractive photography and suspension traction photography were used to determine the patient's spine elasticity as well as the largest orthopedic angle of the patient during the operation. MRI scans and CT scans of the spine were performed before the operation to determine whether there were lesions with or without neural structures such as spinal cord cavities and cauda equina and to determine the actual rotation angle of the pedicle of the rotational deformity. The minimum diameter of the pedicle lays the foundation for the determination of intraoperative positioning and screw insertion angle. At the same time, pulmonary function tests, somatosensory evoked potentials, and action evoked potentials were performed to determine whether there was damage to other organs. Before the operation, conventional spinal traction therapy was used to relax the small joints of the cervical spine, and the adaptability of the nerves in each group to stretching was observed. Patients in the control group received traditional pedicle screw internal fixation. Patients in the study group were treated with 3D printing-assisted pedicle screws for 3D fixation [3].

### 2.2. Observation Indicators

The visual analog scale (VAS) score, Japanese Orthopaedic Association Evaluation Treatment (JOA) score, quality of life score, scoliosis Cobb's angle, pelvic incidence-lumbar lordosis (PI-LL, Table 1), and postoperative complications were compared between the two groups.

### 2.3. Statistics

The data in this experiment were analyzed by SPSS21.0 (SPSS, Chicago, IL, USA), in which the count data (*n*, %) were analyzed by *χ2* test, and the measurement data (‾*x* ± SD) were analyzed by *t*-test. *P* < 0.05 (two-sided) represents statistical significance.

## 3. Results

### 3.1. Baseline Data of Patients

A total of 160 eligible patients (78 and 82 in the control group and the study group, respectively) were retrieved. The average age of patients in the control group was (56.96 ± 5.02) years old, and that in the study group was (56.51 ± 6.36) years old. There were no differences in gender, age, and past medical history between the two groups (*P* > 0.05 for all comparisons). The clinical characteristics of the patients were shown in Table 2.

### 3.2. Comparison of Cobb's Angle, Pelvic Projection Angle, and PI-LL before and after Surgery

There was no significant difference in scoliotic Cobb's angle (20.58 ± 2.03 vs 20.47 ± 2.10) or PI-LL (35.51 ± 0.56 vs 35.23 ± 0.49) between the study group and the control group before surgery (*p*=0.564 and 0.826, respectively). After surgery, Cobb's angle of scoliosis (5.10 ± 0.32) and PI-LL (13.92 ± 0.37) in the study group were lower than those before surgery (*P* < 0.05, Table 3).

### 3.3. Comparison of VAS Score and JOA Score before and after Surgery

No significant differences existed in the VAS score (7.58 ± 2.13 vs 7.47 ± 2.25) or JOA score (12.57 ± 0.38 vs 12.26 ± 0.50) between the study group and the control group (*p*=0.564 and 0.826, respectively) before surgery. After surgery, there were significant differences in the VAS score (3.10 ± 0.18 vs 4.41 ± 0.56) and JOA score (23.42 ± 0.36 vs 19.50 ± 0.51) between the study group and the control group (*P*=0.005 and *P* < 0.001, respectively, Table 4).

### 3.4. Quality of Life Comparison

Before surgery, there were no significant differences in the social function (63.80 ± 3.62 vs 65.61 ± 2.80), physical function (64.23 ± 5.51 vs 64.35 ± 5.08), role function (67.00 ± 6.02 vs 66.53 ± 6.25), or cognitive function (62.97 ± 4.28 vs 64.33 ± 3.14) between thestudy group and the control group (*P*=0.245, 0.051, 0.102, and 0.067, respectively). After surgery, there were significant differences in the social function (82.84 ± 1.15 vs 79.13 ± 3.20), physical function (84.50 ± 3.80 vs 75.44 ± 4.26), role function (83.30 ± 5.38 vs 76.82 ± 6.34), and cognitive function (80.61 ± 4.85 vs 74.35 ± 3.52) between the study group and the control group (*P*=0.001, 0.005, 0.005, 0.001, respectively, Table 5).

### 3.5. Postoperative Complications Comparison

There was a significant difference in the total incidence of postoperative complications between the study group and the control group (*P*=0.001, Table 6).

## 4. Discussion

Degenerative scoliosis occurs through degenerative changes without pre-existing spinal deformity, and it is generally more common in older age groups. It is presented with asymmetric disc space collapse and facet degeneration followed by lateral and/or rotational sliding [7]. This condition, which results in loss of lumbar lordosis as well as sagittal malalignment, will inevitably lead to poor clinical outcomes. Progressive low back pain as well as symptomatic lumbar spinal stenosis are more common in patients with new-onset scoliosis, along with neurogenic claudication or radiculopathy [8, 9]. Generally, symptoms such as progressive clinical deformity and sagittal imbalance will appear later in this group of patients. The treatment of such diseases is complex and based on different pathophysiological and clinical manifestations, with examples of physical therapy and analgesics for many years [10]. Surgical therapies include complex instrumental fusion or simple laminectomy, which are invasive and may have potential complications [11].

About 90% of those patients mainly present with pain, muscle fatigue, and spasticity of scoliosis causing diffuse and axial low back pain in most patients. Judging from the fluoroscopy-guided articular surface injection, all of these people have low back pain due to articular surface degeneration [12, 13]. The disease is characterized by asymmetric disc space and joint degeneration. In this group, there is “hip rib” pain and/or dysfunction due to sagittal imbalance, which is a chronic condition. In the clinical evaluation of such patients, the key is to correctly understand the causes of their pain. Degenerative scoliosis is a complex, multifactorial process that develops over time, so there are many possible etiologies. Pain may be related to major leg joint deformity progression and dysfunction, nerve damage, or degenerative arthritis.

Pedicle screw fixation is aided by 3D printing [14]. The three columns of the spine have a strong control force, and the internal fixation device is tightly mounted to the bone, thereby generating a strong correction force [15, 16]. Suk conducted a retrospective analysis of scoliosis using the pedicle screw technique [17] and found that compared with hook fixation, pedicle screws treated more main thoracic curvature cases (55.8% vs 51.7%). The incidence of postoperative defects was 5.7% and 10.6% in screw therapy and hook therapy, respectively. The postoperative lumbar curvature correction rate was 54.9% and 46.9% in the pedicle screw group and hook fixation group, respectively. In addition, pedicle screws can increase the control of the apical vertebra with maximum rotational deformity, therefore reducing splaying and compression. Studies have shown that directly acting on the spine can not only achieve correction in the coronal plane and sagittal plane but also reconstruct normal anatomy in the transverse plane [18, 19]. However, the anatomy of the thoracic pedicle limits its widespread use. Rampersaud et al. established a morphological model using normal thoracic vertebrae specimens and showed that the implanted screws on the pedicle of the thoracic vertebra had only 1 mm of parallel displacement and 5° of angular offset. When scoliosis occurs in the spine, the angle and transverse diameter of the pedicle will inevitably change due to the rotation and wedge deformation of the vertebral body itself. Therefore, the preoperative image preparation work is to determine the actual angle of the pedicle, the minimum diameter of the pedicle, the relationship between the pedicle and the transverse process, and the distance between the needle insertion site and the anterior edge of the vertebral body for the correction operation. The selection of positioning, entry angle, and implant provides an important reference to improve the accuracy of screw placement [20]. Simultaneous intraoperative EMG and endoscopy are key to preventing screw penetration of the inner wall of the pedicle. In this study, the patients who underwent pedicle screw 3D correction surgery had better treatment effects and fewer postoperative complications, showing that pedicle screw 3D correction surgery had obvious advantages.

To sum up, 3D printing-assisted pedicle screw 3D correction surgery provides a powerful 3D correction force with reliable effect and few complications, and is effective in dealing with degenerative scoliosis.

## Figures and Tables

**Table 1:** Observation Indicators in the present study.

VAS score [4]	0 is the best, the patient has no pain
	1–3 points or less is mild pain that can be tolerated
	4–6 points: The pain is more severe, and the patient's sleep is slightly affected
	7–10 points are unbearable severe pain, the patient cannot sleep, which seriously affects normal life
JOA score [5]	Subjective symptoms
	Clinical signs
	Limitation of daily activities
	The total score is 29 points, a higher score represents a better function
Quality of life score [6]	Cognitive
	Role
	Social
	Physical
	The total score is 100 points. A higher score represents a better life quality

**Table 2:** General information of included patients.

General information	Study	Control	*t*/*χ2*	*P*
*n*	82	78		
Age	56.51 ± 6.36	56.96 ± 5.02	1.812	0.074

Gender			0.202	0.653
Male	44	40		
Female	38	38		

Nationality			1.566	0.211
Han	68	70		
Others	14	8		

Congenital spine disease			0.201	0.654
Yes	0	0		
No	82	78		

**Table 3:** Comparison of scoliotic Cobb's angle and PI-LL between two groups.

Group	Scoliosis Cobb's angle		PI-LL	
	Before	After	Before	After
Study (*n* = 82)	20.58 ± 2.03	5.10 ± 0.32	35.51 ± 0.56	13.92 ± 0.37
Control (*n* = 78)	20.47 ± 2.10	5.91 ± 0.43	35.23 ± 0.49	13.10 ± 0.33
*t*	1.673	12.274	1.538	8.379
*P*	0.564	0.005	0.826	<0.001

**Table 4:** VAS scores and JOA scores comparisons.

Group	VAS score		JOA score	
	Before	After	Before	After
Study (*n* = 82)	7.58 ± 2.13	3.10 ± 0.18	12.57 ± 0.38	23.42 ± 0.36
Control (*n* = 78)	7.47 ± 2.25	4.41 ± 0.56	12.26 ± 0.50	19.50 ± 0.51
*t*	1.673	12.274	1.538	8.379
*P*	0.564	0.005	0.826	<0.001

**Table 5:** Quality of life comparison.

Group	Social function		Physical function		Role function		Cognitive function	
	Before	After	Before	After	Before	After	Before	After
Control	65.61 ± 2.80	79.13 ± 3.20	64.35 ± 5.08	75.44 ± 4.26	66.53 ± 6.25	76.82 ± 6.34	64.33 ± 3.14	74.35 ± 3.52
Study	63.80 ± 3.62	82.84 ± 1.15	64.23 ± 5.51	84.50 ± 3.80	67.00 ± 6.02	83.30 ± 5.38	62.97 ± 4.28	80.61 ± 4.85
*t*	2.019	15.943	1.631	12.055	1.461	13.325	2.130	10.142
*P*	0.245	0.001	0.051	0.005	0.102	0.005	0.067	0.001

**Table 6:** Comparison of postoperative complications between the two groups of patients (*n*, %).

Group	Bleeding	Infect	Pulmonary embolism	Total incidence
Study (*n* = 82)	3 (3.66)	2 (2.44)	0 (0)	5 (6.10)
Control (*n* = 78)	4 (5.12)	3 (3.85)	2 (2.56)	9 (11.53)
*χ2*				8.310
*P*				0.001

## Data Availability

The data used in this study is available from the corresponding author upon reasonable request.
